RETRACTED

# Analysis of the Efficacy of Multidrug Combination Chemotherapy Regimens for Osteosarcoma and the Management of Chemotherapeutic Reactions

**DOI:** 10.1155/2022/6510429

**Published:** 2022-08-25

**Authors:** Dawei Tian, Kun Feng, Xiaobao Wu, Chao Gao, Lixin Hu

**Affiliations:** ^1^Department of Orthopedics, Sinopharm Dongfeng General Hospital of Hubei University of Medicine, Shiyan 442000, Hubei, China; ^2^Department of Postgraduate Training Base, Sinopharm Dongfeng General Hospital of Jinzhou Medical University and Hubei University of Medicine, Shiyan 442000, Hubei, China

## Abstract

**Purpose:**

To analyse the efficacy of high-dose methotrexate + adriamycin + cisplatin (HD-MTX + ADR + PDD, MAP) regimens applied to osteosarcoma and the pretreatment and resolution of chemotherapeutic reactions.

**Methods:**

The clinical data of 21 patients with osteosarcoma in our hospital from January 2015 to January 2018 were retrospectively analysed. All patients were treated with the MAP protocol, 21 days for 1 cycle, and treated with artificial joint replacement or amputation after 3∼4 cycles of treatment. The tumour tissue necrosis rate, limb preservation success rate after treatment, and chemotherapy response during chemotherapy were counted and analysed for all patients. A local recurrence rate, a distant metastasis rate, and an overall survival rate were recorded during the 3-year follow-up period.

**Results:**

After treatment, the percentage of tumour tissue necrosis ≥90% was 85.71% (18/21) and the percentage of successful limb preservation was 57.14% (12/21) in 21 patients with osteosarcoma. During chemotherapy, all 21 patients with osteosarcoma experienced various degrees of chemotherapy reactions, mainly bone marrow suppression of 100% (21/21), gastrointestinal reactions of 100% (21/21), liver function impairment of 66.67% (14/21), and cardiotoxicity of 52.38% (11/21), all of which improved and completed treatment after treatment. During the 3-year follow-up period, the 21 patients with osteosarcoma had a local recurrence rate of 9.52% (2/21), a distant metastasis rate of 28.57% (6/21), and an overall survival rate of 80.95% (17/21).

**Conclusion:**

With stringent protection and relief measures, patients with osteosarcoma treated with the MAP regimen have promising near-term outcomes, with high survival rates over 3 years and tolerable chemotherapy responses. The clinical trial is registered under L2015093.

## 1. Introduction

Osteosarcoma is a primary malignant tumour of bone tissue, which originates from the mesophyll tissue of undifferentiated bone. The main feature is the presence of spindle-shaped stromal cells that produce bone-like tissue, and fibrous and cartilaginous tissue can also be seen in the tumour tissue. It can occur anywhere in the body, with 80% to 90% occurring in long tubular bones, commonly in the actively growing distal femur, proximal tibial epiphysis, and, to a lesser extent, the proximal humerus, accounting for approximately 11.7% of primary bone tumours in humans [1, 2]. Osteosarcoma mostly occurs in young and middle-aged people aged 15 to 25 years old. Clinical manifestations include swollen and painful limbs, high local temperature, varicose veins, mental decrepitude, weight loss, loss of appetite, motor impairment, and other typical symptoms, showing rapid progression, poor treatment effect, and high mortality rate [3, 4].

RETRACTED

Currently, preoperative neoadjuvant chemotherapy combined with surgical resection is more common in the treatment of osteosarcoma, with a five-year tumour-free survival rate of 50–70% and a local recurrence rate of 5–10% in patients [5, 6]. However, for patients with lung metastases present at the time of initial diagnosis, the 2-year tumour-free survival rate is only 28% if there are ≥3 metastases [7]. In recent years, the recommended drugs for neoadjuvant chemotherapy in osteosarcoma are high-dose methotrexate (HD-MTX), adriamycin (ADR), cisplatin (PDD), and ifosfamide (IFO), administered mainly in combination or in sequential doses, which can significantly improve the prognosis of patients with nonmetastatic osteosarcoma [8]. However, in view of the late development of chemotherapy for osteosarcoma in China, chemotherapy for osteosarcoma mostly refers to foreign chemotherapy schemes. Clinical research [9] shows that the efficacy of these schemes applied to domestic patients is limited. Therefore, it is necessary to explore and formulate chemotherapy schemes suitable for domestic patients.

This study analyses the efficacy of the application of the HD-MTX + ADR + PDD (MAP) regimen for the treatment of osteosarcoma and the pretreatment and resolution of chemotherapeutic reactions. Details are as follows.

## 2. Materials and Methods

### 2.1. General Data

Retrospective analysis of the clinical data of 21 patients with osteosarcoma in our hospital from January 2015 to January 2018: inclusion criteria: ① pathologically confirmed untreated primary osteosarcoma. ② No previous history of tumours. ③ Stages I and II, as determined by Enneking staging. ④ No other conditions that might interfere with chemotherapy. ⑤ The patient's clinical profile was complete. ⑥ All patients were treated in our hospital with the MAP protocol combined with prosthetic arthroplasty or amputation. The general clinical information of the 21 patients with osteosarcoma is shown in Table 1.

RETRACTED

### 2.2. Chemotherapy Regimens

MAP regimen: MTX (Yue Kang Pharmaceutical Group Co., Ltd., Approval No. H20113120) at 10–12 g/m^2^ was administered intravenously for 6 h on the first day and 6 hours after the intravenous infusion of MTX; 25 mg of calcium folinate (Jiangsu Hengrui Pharmaceutical Co., Ltd., Approval No. H20000584) was injected intramuscularly for rescue, once every 6 hours for a total of 14–16 times; ADR (Hanhui Pharmaceutical Co., Ltd., Approval No. H33021980) at 50 mg/m^2^ was applied in 2 divided doses on days 6 and 7; PDD (Qilu Pharmaceutical Co., Ltd., Approval No. H37021357) at 80–100 mg/m^2^ was applied in 2 divided doses on day 6 and 7; intravenous rehydration was 3,000 ml per day during MTX treatment and the patient was advised to drink plenty of fluids to promote adequate hydration; the patient was also given 5% sodium bicarbonate (Shandong Shenglu Pharmaceutical Co., Ltd., Approved No. H37021234) 250 ml intravenously twice/day, and took sodium bicarbonate tablets (Hebei Sangshi Pharmaceutical Co., Ltd., Approved No. H13022430) of 1.0 g orally 3 times/day and allopurinol (Chongqing Qingyang Pharmaceutical Co., Ltd., Approval No. H50020548) of 100 mg orally 3 times/day to alkalinize the urine and supplemented with acid-suppressing (e.g., proton pump inhibitor) antiemetic drugs (e.g. metoclopramide and 5-hydroxytryptamine inhibitor) orally, and urine was monitored daily to maintain pH between 7 and 9 for a total of 5 d. During the treatment of PDD and ADR, at least 2500 ml of intravenous fluids were replenished every day, diuretics were used, and blood routine and liver and kidney functions were tested on the 5th day after MTX chemotherapy and the 2nd day after all chemotherapies. 21 days was one cycle. After 3∼4 cycles of treatment, the lesion location was reexamined. After MRI and plain film evaluation, artificial joint replacement or amputation was performed.

### 2.3. Assessment Indicators

The tumour tissue necrosis rate, limb preservation success rate after treatment, and chemotherapy response during chemotherapy were counted and analysed for all patients. Tumour tissue necrosis rate: this was determined according to the Huvos rating system [10], and through the pathological examination of osteosarcoma, the tumour tissue necrosis rate (the largest cross-section of the tumour after decalcification of the postoperative specimen was taken, and the two pathologists jointly judged) and the limb salvage success rate were used to evaluate the overall treatment effect. If the patient had ≥90% tumour tissue necrosis on postoperative pathology, the original regimen of chemotherapy was continued for 3 cycles, if <90%, then high-dose MTX and PDD combined with IFO relief chemotherapy were used instead. Chemotherapy reactions include bone marrow suppression, gastrointestinal reactions, oral ulcers, hepatic and renal impairment, cardiotoxicity, neurotoxicity, and allergic reactions. The grading criteria for chemotherapy drug toxicities 0–IV were determined according to the WHO standards [11].

RETRACTED

Patients' local recurrence rates, distant metastasis rates, and overall survival rates were recorded during the 3-year follow-up period. Local recurrence rate: local recurrence at the primary site of the tumour, usually due to the growth of untreated residual living tumour cells. Distant metastasis rate: the rate of metastasis to the lung, bone, and abdomen. Overall survival rate: follow-up the survival rate of all patients from the beginning of chemotherapy (MAP regimen, surgery) to 1, 2, and 3 years after the end of treatment, including the survival rate with tumour.

### 2.4. Statistical Methods

SPSS 22.0 software was used. Count data were expressed as ratio (%), and the *χ*^2^ test was used for comparison, while the measurement data were expressed as mean ± standard deviation (*x* ± *s*) and compared using the *t*-test. *P* < 0.05 was considered statistically significant.

## 3. Results

### 3.1. Analysis of the Recent Outcome of 21 Patients with Osteosarcoma

After treatment, the percentage of patients with tumour tissue necrosis ≥90% was 85.71% (18/21) in 21 patients with osteosarcoma whose pathological type was common, 14.29% (3/21) in patients with tumour tissue necrosis <90%, 57.14% (12/21) in patients with successful limb preservation, and 42.86% (9/21) in patients with failed limb preservation, as seen in Table 2.

### 3.2. Analysis of Chemotherapy Reactions during Chemotherapy in 21 Patients with Osteosarcoma

During chemotherapy, all 21 patients with osteosarcoma experienced various degrees of chemotherapy reactions, mainly bone marrow suppression of 100% (21/21), gastrointestinal reactions of 100% (21/21), liver function impairment of 66.67% (14/21), and cardiotoxicity of 52.38% (11/21), as seen in Table 3.

### 3.3. Analysis of the Management of Chemotherapy Reactions in 21 Patients with Osteosarcoma

#### 3.3.1. Hematotoxicity

Haematological toxicity appeared 4–5 days after MTX chemotherapy or 7 days after the end of the whole course of treatment. Treatment was mainly by subcutaneous injection of granulocyte-colony-stimulating factor and granulocyte-macrophage colony stimulating factor, and, if necessary, by transfusion of component blood. We add imipenem and cilastatin sodium for injection and fluconazole for grade IV leukopenia with infection or hyperthermia, along with bedside isolation, ultraviolet disinfection, and treatment in a separate ward or transfer to a laminar flow room. Prompt treatment of ordinary patients with bone marrow suppression of grade II or higher was done. Patients with previous myelosuppression of grade III or higher were treated prophylactically 48 hours after the administration of chemotherapy drugs. After 3∼5 days of treatment, the patients recovered gradually, and in severe cases, they recovered to normal in 7∼14 days.

RETRACTED

#### 3.3.2. Gastrointestinal Reactions

Most of them occurred 2–5 days after chemotherapy, vomiting also occurred on the day of administration. Central antiemetic drugs were continuously given until the reaction disappeared, and severe vomiting was temporarily treated with a metoclopramide needle. Patients with frequent diarrhoea were treated with Smecta. Patients with oral ulcers were treated with Kangfuxin gargle, Xilei powder for external use, and compound vitamin B and zinc gluconate tablets orally. Patients with gastrointestinal bleeding were treated with antacids, hemostasis, and blood transfusion. We apply medication promptly after the onset of symptoms and it is cured within 5 days.

#### 3.3.3. Hepatotoxicity

Most of them occurred 2 to 5 days after chemotherapy and were mostly transient liver function abnormalities that recovered quickly after stopping the drug. For those who still had liver damage after stopping the drug, glycine was given continuously to protect the liver and it is cured in 3–6 days.

#### 3.3.4. Cardiotoxicity

It appeared 1 month after chemotherapy. Two of the cases with grade III cardiotoxicity were both sinus tachycardia and one was with T-wave changes. Medication was started after the onset of symptoms and both improved after 2 weeks of treatment with betaloc tablets.

#### 3.3.5. Nephrotoxicity

All cases in this group had mild haematuria and proteinuria, without elevated creatinine or urea nitrogen. All improved after regular review.

#### 3.3.6. Skin Toxicity

The rash appeared on the same day or 3 to 5 days after the drug was administered and was cured 3 to 5 days after antiallergic treatment. Pigmentation appeared in the first month of chemotherapy and gradually faded away about six months after chemotherapy was stopped. Hair loss started 1 month after chemotherapy and could not be graded as all patients were asked to shave their hair at the start of chemotherapy, total hair loss was 100%, and hair regrowth started 1 month after the end of chemotherapy.

#### 3.3.7. MTX Poisoning

Two cases (9.52%) of MTX toxicity were seen in this group, with clinical manifestations appearing 3 days after the use of HD-MTX, and their various complications were managed symptomatically according to the different symptoms described previously. In 2 cases of poisoning, 1 patient had a low, asymptomatic 72-hour MTX blood level exceedance, calcium folinate 15 mg was added at 6-hour intervals, and the blood drug concentration returned to normal after 1 day. In the other case, the 72-hour MTX blood drug concentration exceeded the limit by a large margin, and the symptoms of toxicity were severe, the most serious of which was a degree IV myelosuppression and a degree IV oral mucositis, which prevented the patient from eating for more than a month due to blood oozing from the mucous membrane of the mouth and lips and restricted mouth opening. The patient was treated with intravenous calcium folinate drip until the MTX blood levels dropped to normal and then gradually improved after more than 1 month of symptomatic treatment.

RETRACTED

### 3.4. Analysis of Local Recurrence and Distant Metastasis Rates in 21 Patients with Osteosarcoma during the 3-Year Follow-Up Period

During the 3-year follow-up period, the local recurrence rates of the 21 patients with osteosarcoma were 0.00% (0/21), 4.76% (1/21), and 9.52% (2/21) in years 1, 2, and 3, respectively, and the distant metastasis rates were 4.76% (1/21), 9.52% (2/21), and 28.57% (6/21), as seen in Figure 1.

### 3.5. Analysis of the Survival Rate of 21 Patients with Osteosarcoma during the 3-Year Follow-Up Period

During the 3-year follow-up period, the overall survival rates of the 21 patients with osteosarcoma were 90.48% (19/21), 85.71% (18/21), and 80.95% (17/21) at year 1, year 2, and year 3, respectively, as seen in Figure 2.

## 4. Discussion

In 2009, the annual meeting of the European Society of Clinical Oncology recommended that the recognised effective and commonly used first-line chemotherapeutic agents be MTX, ADR, PDD, and IFO (Class Ib, Evidence Category A) [12]. The efficiency of the above four agents alone is only close to 30%, but the combination of these agents can have a synergistic effect and may result in 100% tumour necrosis in vivo, in addition to reducing drug resistance development [13].

Currently, the clinical use of MTX, ADR, PDD, and IFO in combination with chemotherapy for osteosarcoma can result in a 5-year survival rate of 44–65%, but some patients still have a poor prognosis [14]. In order to identify treatment strategies to improve osteosarcoma and to determine whether patients have a better or worse risk of local recurrence, distant metastases and death are significant. In this study, 21 patients with osteosarcoma were treated with HD-MTX combined with ADR and PDD neoadjuvant chemotherapy. After treatment, 85.71% of the 21 patients with osteosarcoma had a tumour necrosis rate ≥90%, and 57.14% had successful limb salvage. The above indicates that the short-term efficacy of patients is obvious. However, due to the small number of patients and the short observation time, it is necessary to accumulate the number of patients in the future to continue to observe the short-term and long-term efficacy of large samples.

RETRACTED

HD-MTX has a dramatic effect on bone marrow cells, gastrointestinal tract, skin, oral mucosal cells, and hepatocytes, which have a short cell cycle and rapid proliferation rate, and can lead to a variety of adverse reactions such as bone marrow suppression, gastrointestinal reactions, mucositis, oral ulcers, and liver function damage [15, 16], and the mortality of related adverse reactions is about 6% [17]. Therefore, the status of HD-MTX multidrug combined chemotherapy in the treatment of osteosarcoma is controversial. In this study, 21 patients with osteosarcoma were treated with HD-MTX in combination with ADR and PDD under various control measures. During chemotherapy, all patients experienced various degrees of chemotherapy response. From the incidence of chemotherapy reaction, the main manifestations of patients were bone marrow suppression, gastrointestinal reactions, hair loss, liver function damage, and heart damage. In terms of the grade and degree of chemotherapy reaction, with the exception of haematological toxicity, the majority of patients had mildly reversible side effects, and those with grade III or IV toxicity had mainly haematological, some gastrointestinal reactions, and cardiotoxicity, all of whom improved and completed their treatment after effective management. This shows that the safety of patients with osteosarcoma treated with the MAP regimen is guaranteed under strict protection and relief measures. This study also retrospectively evaluated the survival status of 21 patients with osteosarcoma during the 3-year follow-up period and found that the local recurrence rate was 9.52%, the distant metastasis rate was 28.57%, and the overall survival rate was 80.95% in all patients. The results were generally consistent with previous reports.

Most scholars have concluded that pharmacokinetic parameters such as drug blood peak concentration, area under the drug-time curve, elimination rate, and half-life of HD-MTX used in patients with osteosarcoma are closely related to the degree of adverse effects and prognosis of tumour tissue [18–20]. However, the incidence and severity of adverse effects are more complicated in the case of HD-MTX in combination with multidrug chemotherapy. How to ensure the effective blood peak concentration of MTX without affecting the survival rate of patients and how to reasonably use calcium folinate for detoxification have become an important issue in the multidrug combination chemotherapy regimens containing HD-MTX. In this study, for patients whose MTX blood drug concentration was still >0.1 *μ*mol/L at 72 hours, the blood drug concentration was repeated daily until it was <0.1 *μ*mol/L. At the same time, effective detoxification measures had been taken. For those with low MTX blood levels and mild symptoms of poisoning, oral treatment with calcium folinate was administered and the patient's blood drug concentration returned to normal after 1 day; for those with high MTX blood drug concentration and severe symptoms of poisoning, especially those with severe gastrointestinal reactions, treatment with intravenous calcium folinate injection was used until the blood drug concentration returned to normal. The above monitoring of MTX blood drug concentration and the effective rescue of calcium folinate make the incidence of MTX poisoning affecting the course of chemotherapy in this study only 4.76%, and there are no deaths during chemotherapy. It can be concluded that the use of HD-MTX in combination with ADR and PDD neoadjuvant chemotherapy for the treatment of osteosarcoma patients in this study not only ensures the drug blood peak concentration and efficacy of MTX but also does not lead to an increased incidence of MTX toxicity, which is a multidrug combination chemotherapy regimen with both safety and efficacy.

RETRACTED

In summary, the drug toxicities of multidrug combination chemotherapy regimens using HD-MTX-containing chemotherapy are more complex and diverse than those of single-agent HD-MTX chemotherapy, but with stringent protection and relief measures, patients with osteosarcoma treated with the MAP regimen have promising near-term outcomes, with high survival rates over 3 years and tolerable chemotherapy responses.

## Figures and Tables

**Figure 1:** Local recurrence and distant metastasis rates in 21 patients with osteosarcoma during the 3-year follow-up period (%).

**Figure 2:** Survival situation of 21 patients with osteosarcoma during the 3-year follow-up period (%).

**Table 1:** General clinical information of 21 patients with osteosarcoma (*n*, %).

Clinical information	*n*	Percentage
Gender		
Male	12	57.14
Female	9	42.86
Age/years		
＜15	1	4.76
15∼25	18	85.72
＞25	2	9.52
Type of pathology		
Common type	19	90.48
Telangiectatic type	1	4.76
Chondroblastoma-like osteosarcoma	1	4.76
Enneking staging		
I	8	38.10
II	13	61.90
Tumour location		
Upper tibia	10	47.62
Lower femur	6	28.57
Upper femur	3	14.29
Humerus	1	4.76
Upper ulna	1	4.76
Alkaline phosphatase (AKP) levels		
Normal	7	33.33
Rise	14	66.67
Preoperative chemotherapy cycle		
3 cycles	15	71.43
4 cycles	6	28.57

RETRACTED

**Table 2:** Recent outcome of 21 patients with osteosarcoma (*n*, %).

Result	*N*	Percentage
Tumour tissue necrosis		
≥90%	18	85.71
＜90%	3	14.29
Limb preservation results		
Success	12	57.14
Failure	9	42.86

**Table 3:** Chemotherapy reactions during chemotherapy in 21 patients with osteosarcoma (*n*, %).

Chemotherapy reactions	Grade				
	I	II	III	IV	Total
Hematotoxicity					
Leukopenia	1 (4.76)	5 (23.81)	9 (42.86)	6 (28.57)	21 (100.00)
Decreased haemoglobin	2 (9.52)	4 (19.05)	11 (52.38)	4 (19.05)	21 (100.00)
Decreased platelets	1 (4.76)	1 (4.76)	5 (23.81)	7 (33.33)	14 (66.66)
Gastrointestinal reactions					
Nausea, vomiting	6 (28.57)	9 (42.86)	3 (14.29)	3 (14.29)	21 (100.00)
Oral mucositis	6 (28.57)	3 (14.29)	4 (19.05)	1 (4.76)	14 (66.67)
Gastrointestinal bleeding	3 (14.29)	1 (4.76)	1 (4.76)	0 (0.00)	5 (23.81)
Diarrhoea	1 (4.76)	1 (4.76)	0 (0.00)	0 (0.00)	2 (9.52)
Hepatotoxicity					
Elevated alanine transaminase	6 (28.57)	8 (38.10)	0 (0.00)	0 (0.00)	14 (66.67)
Cardiotoxicity					
Cardiac damage	6 (28.57)	3 (14.29)	2 (9.52)	0 (0.00)	11 (52.38)
Nephrotoxicity					
Haematuria, proteinuria	4 (19.05)	1 (4.76)	0 (0.00)	0 (0.00)	5 (23.81)
Skin toxicity					
Rash	4 (19.05)	2 (9.52)	0 (0.00)	0 (0.00)	6 (28.57)
Pigmentation	2 (9.52)	1 (4.76)	0 (0.00)	0 (0.00)	3 (14.29)

## Data Availability

The data to support this study are available at reasonable request to the corresponding author.
